This article has been retracted.

# College English Multimodal Teaching Based on Digital Information Technology

**DOI:** 10.1155/2022/2911215

**Published:** 2022-07-30

**Authors:** Dan Wu

**Affiliations:** School of Foreign Languages, The College of Post and Telecommunication of WIT, Wuhan 430073, Hubei, China

## Abstract

In the era of in-depth application of knowledge technology in the field of education, the teaching mode combining school English teaching and network data technology is widely used in school English education. Teaching resources have become electronic resources under the influence of digital information technology. However, English teaching often ignores all aspects of English ability, so there are still shortcomings in English teaching. The role of information technology makes a single English teaching text model unable to meet the needs of scholars. In recent years, multimodal events have enriched the expression of language input and output content, which is in line with the learning needs of current students. Therefore, under the premise of digital information technology, this paper constructs a multimodal English teaching model from the aspects of multimodal English teaching resources, multimodal English teaching activities, and multimodal English teaching analysis. It aims to mobilize the enthusiasm of scholars to learn English from various aspects and build a multimodal teaching mode of English for teachers supported by digital data technology. Therefore, the experiment shows that the multimodal teaching mode of college English based on digital information technology proposed in this paper will mobilize the enthusiasm of students to learn in a comprehensive way. It greatly improves students' English performance, promotes the development of students' autonomous learning ability and comprehensive language ability, and improves the quality of English teaching by 20%.

## 1. Introduction

At present, English teaching has been integrated with network information technology. In particular, English teaching in colleges and universities has been deeply integrated with multimedia teaching. Teachers basically use multimedia teaching mode in class [1]. However, although this teaching mode has made some progress with the traditional teaching mode, it still continues the drawbacks of the traditional teaching mode, especially the students' enthusiasm in the classroom and learning initiative. However, it still did not change the attitude of students towards English learning, and the subjective initiative of students and the dominant position of the classroom were not brought into play [2]. This makes the students' autonomous learning ability and comprehensive English language ability still cannot be significantly improved. English teaching also lacks activities with language communication, which exacerbates the tendency of “cramming” and “one talk,” thus limiting students' creativity. However, teachers in colleges and universities still do not pay attention to whether there is a problem with their own teaching methods. They still adopt the traditional teaching mode, and only convert the textbooks into multimedia display, and the teaching concept has not changed. In order to change this phenomenon in English teaching and stimulate students' initiative in English language learning and creativity in the classroom, it is necessary to change the way of English teaching.

In order to improve the teaching quality of English in colleges and universities, many scholars have conducted research on the corresponding teaching mode. Among them, Wang P started from the concept of multimodal teaching, introduced the multimodal media system and theory, and constructed a multimodal adaptive teaching mode based on multimodal reading and writing, knowledge reading, and cognitive construction. This provides a reference for improving students' English learning ability and teachers' teaching quality [3]. But his research lacks real-data validation. Liu and Jiang [4] mentioned the issues existing within the learning of “PHP website development technology” in class. He discerned the issues of single ancient teaching ways and single English teaching ways in colleges. He additionally explained the practicability and necessity of deepening the reform of English info teaching by faculties in universities [4]. Wen J expounded the appliance and thought of the multi-interactive teaching mode and introduced the connected learning theory. He verified the effectiveness of the multi-interactive teaching model in school English teaching through elaborated teaching experimental style and comparative analysis of teaching results [5]. But his research lacks theoretical support and is not very convincing. Chen et al. [6] studied the flipped classroom teaching mode of college English based on the O2O teaching system. He explored teaching modes related to students' autonomous learning ability, and further constructed a classroom teaching mode scheme with teaching guidance suitable for English teaching. The experimental results demonstrate the effectiveness of the proposed model and method [6]. His research did not elaborate on the construction process of the proposed model, and it was difficult to understand. Li [7] proposed that the net and server terminals extend education on the far side the schoolroom. On this basis, he mentioned the development of a mixed teaching mode of faculty English supported trendy academic technology and engineering [7]. There are no specific experimental data for his research. Diao and Hu [8] analyzed the complexity of deep learning and the application of multimodal object recognition in English education systems. He proposed that the large-scale application of multimedia technology in college English classrooms is conducive to the construction of a real language environment. The simulation results show that 84% of students believe that the multi-modal teaching mode is closer to life [8]. His research has not conducted in-depth discussions on deep learning and the research lacks depth. Although their research has certain reference value for English teaching, they all have certain deficiencies. Therefore, this paper makes a new exploration of English teaching mode on the basis of their research. Digital information technology has enriched the display form of teaching resources and improved the fun of teaching. Students' interest in learning can be significantly improved [9].

The English multimodal teaching discussed in this paper can improve the shortcomings of the previous teaching mode and give full play to the students' autonomous learning ability. In particular, it promotes a substantial improvement in English listening and speaking skills. The combination of multimodal teaching mode and digital information technology will reshape teachers' teaching concepts and change teachers' teaching strategies. It transforms teachers' teaching strategies from the ancient teaching mode to the integrated teaching mode of “teaching, learning, and doing.” In addition, the multimodal English teaching method can give full play to the students' initiative, so that the students' English ability can be developed in a balanced way. It stimulates creativity in English learning and improves students' interest in English learning.

This paper has the following innovations in the research on the multimodal teaching mode of college English based on digital information technology: (1) compared with the traditional teaching mode, multimodal teaching can classify the learning types of students. And it enables students to interact with the external environment and stimulate students' subjective initiative in an all-round way. (2) The combination of digital information technology and multimodal teaching mode can combine the advantages of both. It combines a variety of teaching methods to give full play to the advantages of a variety of teaching methods. (3) Digital information technology can enrich the presentation form of teaching resources and make the classroom full of modern atmosphere and a learning atmosphere.

## 2. Methods of College English Multimodal Teaching

### 2.1. Digital Information Technology and Teaching

Digitization is to transform a lot of complex and changeable information into measurable numbers and data, and then, process these information in a unified manner inside the computer [10]. The information age has caused the rapid expansion of information, and it has been difficult for humans to process massive amounts of information. Now, we are in the era of informationization, and the amount of information has increased dramatically. It is a very cumbersome to process these massive amounts of information manually, so the use of computers to process massive amounts of information can greatly improve the efficiency of information processing and save a lot of human input [11]. Therefore, to process information with a computer, it is necessary to digitize the information in order to be able to process these huge and complex information. The application areas of information digitization are shown in Figure 1:

Information technology includes sensor technology, communication technology, etc., Digital information technology digitizes received information on the basis of these technologies [12]. At present, college teaching has been integrated with network information technology. For example, multimedia displays, pictures, videos, and other teaching resources can be found on the Internet, which are all realized through communication technology and network information technology [13]. However, it is necessary to display teaching resources in new formats such as videos and pictures, and someone needs to tamper with the teaching materials behind the network. Only when it is transformed into pictures and video information can real multimedia teaching be realized. Therefore, it is necessary to convert teaching resources into data information and transmit it to the network, which requires a series of conversions. It sets the source teaching materials that need to be converted into digital information as follows:

(1) $$\begin{array}{c} r=\left\{r_{1},r_{2},r_{3},...,r_{n}\right\}. \end{array}$$

All the source teaching resources will be passed to the network layer of the first layer through sensing technology. Of course, the information of the network layer of the first layer is still presented in the form of source information, so the sensing technology only perceives the source information and transmits the source information to the network. The information conversion process diagram is shown in Figure 2.

It can be seen from the Figure 2 that the sensing area of the device in the sensing technology has four nodes: *A*, *B*, *C*, and *D*. Each node has a communication network, which transmits the source information to the information transformation area step by step. These nodes can be divided into distributed and centralized categories. Distributed category does not require high sensor performance, while centralized category is the opposite [14]. Because the amount of data *Q* circulated by the nodes of the sensing device is limited, then, the amount of data from the source data to each node is as follows:

(2) $$\begin{array}{c} Q_{A}=\sum_{n}^{v}r*\phi . \end{array}$$

Then, the first centralized node will be formed at the second node, and the number of source information of the first centralized node is as follows:

(3) $$\begin{array}{c} Q_{B}=\sum_{n}^{v}r*\phi +\sum_{n}^{v}Q_{A}. \end{array}$$

In the above formula, *v* is the transmission speed of the communication network, and *n* represents the number of types of source information to be transmitted by the sensor technology. And *ϕ* is the parallel matrix of the source information in the transmission process, and its form is as follows:

(4) $$\begin{array}{c} \phi =\left[\begin{array}{ccc} A & \cdots & B\\ r_{1} & r & r_{n}\\ C & \cdots & D \end{array}\right]. \end{array}$$

For this reason, the second centralized node is the third distributed node, and the number of source information is as follows:

(5) $$\begin{array}{c} Q_{C}=\left(\sum_{n}^{v}r*\phi +\sum_{n}^{v}Q_{A}Q_{B}\right)*s. \end{array}$$

In the above formula, because the amount of information in the sensing area is getting larger and larger, the information transmission in the sensing area takes time, and *s* represents the transmission time. Therefore, the number of source messages for the last transfer node is as follows:

(6) $$\begin{array}{c} Q_{D}=\left(\sum_{n}^{v}r*\phi +\sum_{n}^{v}Q_{A}\frac{Q_{B}}{Q_{C}}\right)*s. \end{array}$$

So, the total amount of data transmitted to the first network layer of the translation area is as follows:

(7) $$\begin{array}{c} Q=Q_{D}*v*s*\phi . \end{array}$$

Under the induction of sensing technology, it transmits the required resources to the network little by little. In order to better store and process this information, it will be digitized in the intermediate conversion area. In the area of information digitization transformation, the second layer of network is the mapping layer, and the last layer is the information that has become digitized, then the digitized information can be expressed as follows:

(8) $$\begin{array}{c} y=\left\{y_{1},y_{2},...,y_{n}\right\}. \end{array}$$

In the information digitization area, there is an activation function in the mapping layer whose form is as follows:

(9) $$\begin{array}{c} f\left(t\right)=\frac{1-\exp\;\left(-t\right)}{1+\exp\;\left(-t\right)}. \end{array}$$

This activation function is the key to realize the digitization of information. During the transformation, the source information will be continuously encoded and transformed. From the first-layer network to the second-layer network, that is, into the mapping layer, the number of source information resources will become

(10) $$\begin{array}{c} t_{1}=\sum_{n}r_{1}j_{1}^{v_{1}}*s,\\ t_{2}=\sum_{n}r_{2}j_{2}^{v_{2}}*s+t_{1},\\ t_{n}=\sum_{n}r_{n}j_{n}^{v_{n}}*s+\left(t_{1}+t_{2}+...+t_{\left(n-1\right)}\right), \end{array}$$

*j* is the threshold of the network in transition. When the source information is input to the second layer, there is also a process of coding. This code refers to encoding. Each type of source information is encoded for better categorization. It sets the code to *M*, and the principle of coding is as follows:

(11) $$\begin{array}{c} r⟶\frac{v}{s}M*r⟶t. \end{array}$$

So, at the second network layer, the digitization of the source information has already been converted to half. The information it inputs to the third layer in the second layer will be stored in the network as digital information. The principle of inputting information from the second layer to the third layer is as follows:

(12) $$\begin{array}{c} y_{1}=Mt_{1}=\sum_{n}r*v,\\ y_{n}=Mt_{n}=\sum_{n}r_{n}*v. \end{array}$$

In the second layer, all the information will be most comprehensively transformed through the activation function. The principle is as follows:

(13) $$\begin{array}{c} y=t*f\left(t\right)*\sum_{n}Q. \end{array}$$

Ultimately, all information is stored in the network as digital information. If it needs to be reproduced in the form of the source document, it needs to be decoded step by step. Therefore, a large number of teaching resources on the Internet are stored in major websites in this form, and when teachers and students need teaching materials, they can search online and display them in front of people in the form of source information. The development of digital information technology has changed the traditional teaching mode and brought electronic teaching into the field of human education, but it has also brought new problems to teaching. Digital information technology enables teaching content to be presented in various forms, enriching teaching resources and promoting the sharing of learning resources. However, it has not completely changed the shortcomings of traditional teaching, so it is still necessary to improve the education model on the basis of information education [15].

### 2.2. College English Teaching

College English is a public basic course with non-English major undergraduates as the teaching object, which mainly serves the professional learning needs of college students and the training of professional talents [16]. In order to make learning English better help students work in the professional field, it is necessary to enhance students' English level and improve students' listening, speaking, reading, and writing ability. The development of English proficiency will not solely facilitate students at work [17]. It can be seen that the cultivation of English ability cannot simply improve the skill quality of scholars, but must be combined with the cultivation of humanistic quality. It allows students to understand the cultural characteristics of foreign countries and communicate effectively with the other countries without the aid of external forces. This can effectively improve students' understanding and the mastery of other cultures. This enables them to have stronger international communication skills, thereby enhancing their own competitiveness. In addition to these meanings, English learning is also an inevitable requirement for students to integrate into society [18].

However, because college English is aimed at undergraduate students who are not majoring in English, the English level of students faced by college English teaching is uneven. Therefore, teachers cannot take into account the English learning situation of each student. And university education is based on students' autonomy and their own learning ability. In addition, teachers' English teaching mode also plays an important role in students' English learning career [19]. This school English teaching mode keeps pace with the times. Information technology has also been deeply integrated into English teaching in schools. Multimedia teaching is shown in Figure 3:

Figure 3 shows the current teaching mode of college English. Although it has been integrated with the network information technology, the classroom only displays the textbooks in the form of PPT and still follows the traditional teaching mode. That is to say, the network information education equipment and teaching materials belong to the auxiliary status. Classrooms do not make full use of network information education equipment, and English classrooms are still dull and boring, which makes the quality of teaching still stagnant [20]. It is just that the way of display is different, and teachers have not been able to give full play to the functions of network information education equipment. In addition, it is influenced by the teaching philosophy. The teaching philosophy that teachers uphold is to explain the book knowledge to the students. If the students understand and remember it, they have mastered it. Therefore, in the classroom, the teacher conveys the content of the textbook to the students. Under this educational philosophy, foreign-language classrooms are often dominated by teachers. The teacher explains the content of the textbook to the students without hesitation, from grammar, vocabulary, sentences to paragraphs and tries to make the students understand every word in the textbook [21]. The classroom under this concept does not see the students but only the teachers. They do not see the attention and cultivation of students as human beings, only the instillation of book knowledge. This makes students less motivated in the classroom and even doze off [22]. The impact of the current teaching model is shown in Figure 4:

In addition to the problem of teachers' English teaching methods, there is also the attitude of students towards English learning, especially the contemporary college students who have grown up with informatization. In addition, the dullness of the classroom makes students' autonomous learning ability decline. Under the influence of exam-oriented education, students have become machine dominated by exam-oriented students. When they go to university, students have more free time and relatively few English class hours. Students are prone to inertia and then lose interest in English learning [23]. It is precisely because of the English teaching mode and the students' attitude towards English that the overall teaching quality of college English cannot be improved. Therefore, how to improve the effect of English classroom teaching and make teaching more attractive is an urgent problem to be solved.

### 2.3. The Combination of Digital Information Technology and Multimodal English Teaching

Multimodal teaching means that students can learn through the five senses of sight, hearing, antennae, smell, and taste, and the interaction between various senses and the external environment is a modality. It embodies the advanced teaching method integrating “teaching, learning, and doing”, and the multimodal type can also classify the learning type of students, as shown in Figure 5:

As shown in Figure 5, it can be roughly divided into five types: visual learning students, auditory learning students, tactile learning students, smell learning students, and taste learning students [24]. Compared with the single-linear ancient school English teaching mode supported teacher teaching, multimodal English teaching will take into consideration the kinds of students' learning. It will incorporate static resources and dynamic resources into the teaching method through completely different media, offer students with a full vary of multi-sensory experiences, and stimulate students' multi-level associations. In explicit, the teaching of faculty English covers listening, speaking, reading, and writing. Through multimodal teaching ways, students' enthusiasm for learning will be mobilized negatively. This could provide full play to the dominant position of scholars within the English room by applying of recent digital info technology within the field of education. Academics will use network technology to counterpoint teaching ways, amend teaching ideas, absolutely stimulate students' subjective initiative, and change students to effectively absorb English data.

In addition, students will explain the information within the room, let the scholars learn it by themselves, then, show it within the room with the assistance of network info technology additionally. It is necessary to make English divisions within the room, so as to provide full play to the benefits of multimodal teaching, and in order that students will develop during a comprehensive and balanced manner from listening, speaking, reading, and writing. In particular, oral English needs to be exercised, because traditional education does not have an environment for practicing oral English, and students are reluctant to speak, so the ability to speak English is what needs to be cultivated the most. Therefore, it is necessary to create an English environment to promote students to communicate in oral English, so as to effectively improve their oral ability. In addition, using network information technology, teachers can display pictures and let students describe pictures in English, fully mobilize students' senses such as vision and hearing, so that students can devote themselves to English learning wholeheartedly. The teaching mode combining network information technology and multimodality is shown in Figure 6:

Network technology enables diversified display of teaching content, and multimodal English teaching can give full play to students' five senses to participate in learning, which can greatly improve their English ability. In addition, teachers and students' views improve at the same time, and the quality of English teaching will be effectively improved. Of course, this new teaching mode also requires teachers to select appropriate teaching resources when making multimedia courseware. Teachers use digital network technology to carefully search for teaching resources and establish a correct multimodal English teaching concept. They changed the traditional teaching concept and brought the students' dominant position in the classroom into full play. Students also need to improve their independent learning ability and exert their subjective initiative, take responsibility for their own English learning, and improve the quality and effectiveness of English teaching in both directions. Students also need to correct their attitudes towards English learning and improve their ability to learn independently.

## 3. Experiment and Analysis of the New Multimodal English Teaching System

### 3.1. The Situation of Multimodal English Teaching

In this experiment, two classes were selected from a certain university, and the number of majors in these two classes were the same. Before the test, we made a week of classroom observations of the English classes of the teachers who taught the two classes and recorded the presentation form of the teaching content of the two teachers in the multimodal classroom. Then, the English classroom mode of teacher *A* is shown in Table 1.

The English classroom mode of teacher *B* is shown in Table 2.

From Tables 1 and 2, teacher *A*'s teaching forms are varied, including language, text, video, multimedia, and other network information technologies, giving full play to the role of network info technology in teaching. Teacher *B*'s classroom mode is relatively simple, basically using language, text, and chalkboard modes, which fails to present full play to the role of network data technology. During this week's observation, it can be seen that the students under the leadership of teacher *A* are more enthusiastic about English learning and are active in the classroom. However, teacher *B*'s students are more passive, and classroom discussions are not very active. So, in modern teaching, it is necessary to give full play to the role of network information technology. At the same time, this experiment also compared the learning situation of the students in the two classes, as shown in Figure 7:

It can be clearly seen from (a) in Figure 7 that the grades of students in the class led by teacher *A* are significantly better than those in the class led by teacher *B*. The excellent rate of class A reached 37.5, while the excellent rate of class *B* only reached 20. The good rate of class *A* reached 60, while the good rate of class *B* only reached 47.5. Moreover, it can be seen from (b) that the teaching quality of teacher A is obviously better than that of teacher *B*, and the teaching efficiency of teacher A is better.

### 3.2. The Effect of Multimodal English Teaching

This experiment will take 40 students from teacher *B*'s class as experimental samples. First, it records the English level of the current students in this class, and then, asks teacher *B* to change the teaching mode, fully use digital information technology for teaching, and fully mobilize the enthusiasm of the students. In this experiment, students' English listening, speaking, reading, and writing were tested. The comparison of students' listening and speaking test scores before and after teacher B changed the teaching mode is shown in Figure 8:

From Figure 8, it can be seen that the students' listening and speaking scores have improved as a whole after the implementation of the multimodal teaching model. It is said that the proportion of grades in each stage has increased, and the proportion of students who failed the stage has dropped significantly by about 15%. The comparison chart of the scores before and after the reading and writing test is shown in Figure 9:

From the two graphs in Figure 9, after the implementation of the new teaching model, the proportion of grades within the smart stage and the pass stage has magnified considerably, while the proportion of unqualified reading and writing scores has dropped significantly. Therefore, it is found that multimodal English teaching will considerably improve students' English performance. In order to observe the changes of English teaching in the class under the leadership of teacher *B* more intuitively, it also compared the English teaching effect of the whole class and the overall English performance, as shown in Figure 10:

Figure 10 shows that after the implementation of multimodal teaching, students' English scores have been greatly improved, with only 2.44% of the students failing, and the quality of teaching has also improved by about 20%. It also shows that multimodal teaching has a good effect on the improvement of English performance and teaching quality.

### 3.3. Experimental Summary

From the above experiments, we can see the importance of multimodal teaching by comparing the students in teacher *A* and teacher *B* classes. After the change in teaching mode, students' English scores have been greatly improved, and the improvement rate can reach about 20%. The teaching mode of class *A* is diversified, so the overall performance of students is better. The teaching mode of class *B* is relatively simple, so the grades lag behind that of class *A*. Therefore, the combination of digital information technology and multimodal teaching methods can promote the improvement of English teaching quality.

## 4. Discussion

This paper explores the inner principles of digital information technology. Digitization has occupied an unshakable position in the current information age, so digitization has bit by bit been integrated into people's lives within the development of today's society. The network communication technology in the info technology has already affected all aspects of people's lives, so the digital info technology will further develop in the swift growth of modern science and technology. And with the growth of the field of noopsyche, digital info technology is wide utilized in the sector of intelligence, and then applied to other fields, especially in the field of modern education. Modern education and network information technology are deeply integrated. In particular, college English includes listening, speaking, reading, and writing skills, and the traditional college English education model is no longer suitable for students who grew up in the Internet age. And if students want to develop their English skills in an all-round way, they need to start from the four aspects of listening, speaking, reading, and writing. The use of digital info technology within the room multimodal teaching may be terribly appropriate for the interests of recent students. This makes students additionally impelled to be told and provides full play to their subjective initiative.

Multimodal teaching combined with digital information technology can well promote the display of English teaching content. Of course, this teaching model can also be applied to the teaching of other subjects. Only by transforming teaching resources into specific disciplines and making certain adjustments, the overall teaching quality of colleges and universities can be promoted. What's more, the experiment in this paper also proves that this educational model can stimulate students' interest and motivation in learning. It can greatly improve students' academic performance. Therefore, the multimodal teaching mode has a great practicability and can be widely promoted in the teaching field.

## 5. Conclusions

This paper explores digital information and college English education. There is a big problem in college English teaching. Even if it is combined with network technology, it is still hard to change the defects of college English teaching. Therefore, this paper studies the application of digital information technology and multimodal teaching in English teaching. It is found that the teaching method combining multimodal teaching and digital technology can enrich the display form of teaching resources and give full play to the subjective initiative of students. And the experiments in this paper show that the application of digital information technology and multimodal teaching in college English teaching can greatly improve the quality and efficiency of English teaching. This teaching mode can be widely used in efficient classrooms. However, there are still many deficiencies in this paper for the research on the multimodal teaching of college English based on digital information technology. The authors hope that future research can focus on the shortcomings.

## Figures and Tables

**Figure 1:** Digital application areas.

**Figure 2:** Information transformation process diagram.

**Figure 3:** College English teaching.

**Figure 4:** Impact of teaching models.

**Figure 5:** Student learning types.

**Figure 6:** Teaching mode combining network information technology and multimodality.

**Figure 7:** Comparison of classes led by two teachers: (a) comparison of student performance and (b) comparison of teaching quality.

**Figure 8:** Before and after comparison of listening and speaking test scores. (a) Before implementation. (b) After implementation.

**Figure 9:** Before and after comparison of reading and writing test scores. (a) Before implementation. (b) After implementation.

**Figure 10:** Before and after comparison of teacher *B*'s English teaching. (a) Comparison of performance. (b) Comparison of teaching quality.

**Table 1:** Teacher *A*'s English classroom modality.

The modal class type	Reading	Writing	Grammar	Listening
Language	✔	✔	✔	
Text	✔	✔	✔	
Video	✔			✔
Picture			✔	
Audio		✔		✔
Blackboard	✔		✔	
Multimedia	✔	✔		✔

**Table 2:** Teacher *B*'s English classroom modality.

The modal class type	Reading	Writing	Grammar	Listening
Language	✔	✔	✔	
Text	✔	✔	✔	
Video				
Picture				
Audio				✔
Blackboard	✔		✔	
Multimedia				

## Data Availability

The data that support the findings of this study are available from the corresponding authors upon reasonable request.
